The article "Identification of Nine M6A-Related Long Noncoding RNAs as Prognostic Signatures Associated with Oxidative Stress in Oral Cancer Based on Data from The Cancer Genome Atlas" was retracted in 2023. Reasons: signs of a paper mill; compromised peer review; unreliable results or conclusions.

# Identification of Nine M6A-Related Long Noncoding RNAs as Prognostic Signatures Associated with Oxidative Stress in Oral Cancer Based on Data from The Cancer Genome Atlas

**DOI:** 10.1155/2022/9529814

**Published:** 2022-07-22

**Authors:** Li Shan, Ye Lu, Yihua Song, Xiaoli Zhu, Cheng-Cheng Xiang, Er-Dong Zuo, Xu Cheng

**Affiliations:** ^1^Department of Hematology and Oncology, Soochow University Affiliated Taicang Hospital (the First People's Hospital of Taicang), Jiangsu 215400, China; ^2^Suzhou Medical College of Soochow University/Soochow University Affiliated Taicang Hospital, China; ^3^Department of Stomatology Affiliated Hospital of Nantong University, Nantong University, Nantong, Jiangsu, China

## Abstract

**Objective:**

Although the expression of long noncoding RNAs (lncRNAs) and N6-methyladenosine (M6A) is correlated with different tumors, it remains unclear how M6A-related lncRNA functioning affects the initiation and progression of oral squamous cell carcinoma (OSCC).

**Materials and Methods:**

Gene expression and clinical data were retrieved from The Cancer Genome Atlas. The prognostic value of M6A-related lncRNAs was determined using univariate Cox regression analyses. Gene set enrichment analysis of OSCC patient clusters revealed the pathways that elucidate the mechanism. Furthermore, a risk-based model was established. The difference in the overall survival (OS) between groups, including low-/high-risk groups, was determined by Kaplan-Meier analysis. Relationships among immune cells, clusters, clinicopathological characteristics, and risk scores were explored.

**Results:**

Among 1,080 M6A-related lncRNAs, 36 were prognosis-related. Patients with OSCC were divided into two clusters. T stage and the pathological grade were noticeably lower in cluster 2 than in cluster 1. Epithelial-mesenchymal transition showed greater enrichment in cluster 1. Nine hub M6A-related lncRNAs were identified for the model of risk score for predicting OSCC prognosis. The OS was longer in patients with a low-risk score than in patients with a high-risk score. The risk score was an independent prognostic factor of OSCC and was associated with the infiltration of different immune cells. T stages and the American Joint Committee on Cancer (AJCC) stages were more advanced in the high-risk score group than in the low-risk score group. Finally, expression correlation analysis showed that the risk score is associated with the expression of oxidative stress markers.

**Conclusion:**

M6A-related lncRNAs play an important role in OSCC progression. Immune cell infiltration was related to the risk score model in OSCC and could accurately predict OSCC prognosis.

The article "Identification of Nine M6A-Related Long Noncoding RNAs as Prognostic Signatures Associated with Oxidative Stress in Oral Cancer Based on Data from The Cancer Genome Atlas" was retracted in 2023. Reasons: signs of a paper mill; compromised peer review; unreliable results or conclusions.

## 1. Introduction

Approximately 405,000 new oral cancer cases are reported worldwide annually, with the highest incidence reported in Sri Lanka and India [1, 2]. According to the International Classification of Diseases, oral cancer can be categorized into cancers of the tongue, lip, gum, upper jaw, sublingual space, hard palate, buccal mucosa, and retromolar area. The ratio of the number of cases of oral squamous cell carcinoma (OSCC) to those of other types of oral cancer is almost 90% [2, 3]. OSCC has multiple risk factors, primarily smoking, drinking, chewing betel nut, and human papillomavirus infection [4, 5]. Early diagnosis of OSCC is difficult. As a result, the rate of cure is low and the mortality rate is high, which places a heavy burden on individuals and societal economies.

Research on the induction and progression of OSCC at the molecular level is particularly important owing to a lack of biomarkers for early OSCC prognosis and diagnosis. The present study focused on the screening of prognostic biomarkers for OSCC.

N6-Methyladenosine (M6A) epigenetically modifies RNA molecules. M6A can affect tumor progression by inducing suppressor genes and regulating oncogene expression in tumorigenesis and subsequent tumor development. The M6A regulators are controlled by regulatory proteins with methyltransferase activity (“writers”), signal transducers (“readers”), and demethylases (“erasers”) [6]. M6A is related to the induction and development of hepatocellular carcinoma, cervical cancer, breast cancer, and OSCC [7, 8]. Linear RNAs spanning more than 200 nucleic acids are long noncoding RNAs (lncRNAs) and do not encode proteins. lncRNAs affect gene expression at the transcription and posttranscription levels. The degree of tumor malignancy is strongly associated with the dysregulation of lncRNAs [9]. lncRNAs play significant roles in the progression of OSCC [10]. For example, the level of expression of the HOX transcript antisense intergenic RNA (HOTAIR) is related to the tumor size, AJCC stage, and prognosis of OSCC [11]. RNA1, known as the epidermal growth factor receptor antisense (EGFR-AS1), is strongly upregulated in cervical squamous cell carcinoma and is considered a biomarker of OSCC [12]. Findings from the latest research suggest that lncRNAs are responsible for regulating the modification of M6A and consequently the development of cancers, including gliomas and liver cancer [13, 14]. Meanwhile, the mechanism underlying the action of M6A in the dysregulation of lncRNAs in tumor cells and the process by which M6A-related lncRNAs promote the initiation and progression of OSCC remain elusive. GSEA results showed that the signature may be related to oxidative stress. Information about how M6A-related lncRNAs are responsible for the initiation and progression of OSCC can aid the identification of new biomarkers and therapeutic targets.

The article "Identification of Nine M6A-Related Long Noncoding RNAs as Prognostic Signatures Associated with Oxidative Stress in Oral Cancer Based on Data from The Cancer Genome Atlas" was retracted in 2023. Reasons: signs of a paper mill; compromised peer review; unreliable results or conclusions.

Evidence from studies suggests that oxidative stress can increase the infiltration of dendritic cells (DCs) and T cells in the tumor-immune microenvironment and transform cold tumors into hot tumors, thereby promoting a more effective antitumor immune response. Nevertheless, the elimination of oxidative stress increases antitumor immunity and T-lymphocyte infiltration, causing a potent antitumor effect. A previous study showed that, in breast cancer, the removal of oxidative stress in the tumor microenvironment (TME) alleviates immunosuppressive immunogenic cell death induced by oleandrin-based anticancer drugs and induces a more persistent effect on T cells. Collectively, these contradictory results indicate that immunogenic cell death can be induced by modulating oxidative stress to enhance the outcomes of immunotherapy. Hence, further investigations are needed to identify the mechanism underlying oxidative stress and OCSS.

This study investigated M6A-related lncRNAs that could affect OSCC prognosis, based on data from The Cancer Genome Atlas (TCGA). Patients with OSCC were grouped between the two clusters using consensus clustering, and their characteristics were explored. A risk score model was developed for the prediction of OSCC prognosis using nine major M6A-related lncRNAs identified using least absolute shrinkage and selection operator (LASSO) and Cox regression analyses. These M6A-related lncRNAs were determined to contribute significantly to OSCC progression and the risk score model, which could be used precisely for the prediction of OSCC prognosis.

## 2. Materials and Methods

### 2.1. Data Resource

TCGA gene expression data of 371 patients with OSCC and 32 normal individuals (controls) were retrieved from the database website (accessed in April 2021). The data were obtained from patients with OSCC involving the gum, base of the tongue, general parts of the tongue, lips, sublingual space, general parts of the mouth, tonsil, palate, and poorly defined sites in the oral cavity and lip. Corresponding clinical information was available for 368 patients. TCGA-acquired data also included expression data for 23 M6A-related genes, including eight writer genes (METTL16, METTL3, METTL14, RBM15B, WTAP, RBM15, VIRMA, and ZC3H13), 13 reader genes (FMR1, HNRNPC, HNRNPA2B1, IGF2BP3, IGF2BP2, IGF2BP1, LRPRRC, RBMX, YTHDF3, YTHDF2, YTHDC2, YTHDC1, and YTHDF1), and two eraser genes (ALKBH5 and FTO)^A^. The anatomic stage was determined based on the criteria published by the American Joint Committee on Cancer (AJCC) Staging Manual, 8th edition (2017) [15].

The article "Identification of Nine M6A-Related Long Noncoding RNAs as Prognostic Signatures Associated with Oxidative Stress in Oral Cancer Based on Data from The Cancer Genome Atlas" was retracted in 2023. Reasons: signs of a paper mill; compromised peer review; unreliable results or conclusions.

### 2.2. Identifying M6A-Related lncRNAs for OSCC Prognosis, Consensus Clustering, Survival Analysis, and Correlations

Coexpression analysis was performed to screen M6A-related lncRNAs using the Wilcoxon test with the criteria *p* < 0.001 and correlation > 0.4. Following this, the coexpression network was developed using the “igraph” R package. Subsequently, univariate Cox regression analysis was used to identify prognostic M6A-related lncRNAs with *p* < 0.01. Patients with OSCC were grouped into various clusters by consensus clustering depending on the lncRNA expression levels. OS differences in the different clusters were explored using Kaplan-Meier (KM) analysis. Finally, the “pheatmap” and “ggpubr” R plugins were used to examine changes in the expression levels of M6A-related lncRNAs and clinical characteristics between the clusters [16, 17].

### 2.3. Gene Set Enrichment Analysis (GSEA)

To complete the pathway analysis, the GSEA software (v4.0.3) was used. Nominal values (NOM) with (*p* < 0.05) and a false discovery rate (*q* value < 0.25) were both considered statistically significant [18, 19].

### 2.4. Risk Score Model Establishment and Evaluation

A random distribution of patients was performed among the training and test groups using the R plugin “caret.” Major M6A-associated lncRNAs related to patient prognosis in the training group were identified using LASSO Cox analysis. The minimum standard method (evaluation of penalty parameters by at least ten cross-validations) was used to determine the coefficients. After identifying M6A-correlated lncRNAs and their coefficients, a risk score model was established using the following formula:

(1) $$\begin{array}{c} \text{Risk score}=\overset{n}{\underset{i=1}{\sum }}{\text{Coef}}_{i}*x_{i}, \end{array}$$

where Coef_*i*_ = coefficient and *x*_*i*_ = fragments per kilobase of transcript per million (FPKM) value of major M6A-related lncRNAs for OSCC prognosis.

Based on the average risk score, patients were categorized among the high-risk and low-risk score groups. Risk plots, survival analysis, and receiver operating characteristics (ROC) curves were used to assess the efficacy of the risk score model. Additionally, the test group was used to verify the value of the risk score model. Univariate and multivariate Cox analyses revealed the effects of other clinical characteristics and risk scores on the OS. The “survminer” function of R package was used for evaluating the value of the prognostic risk score in a population with various clinicopathological characteristics [20, 21].

### 2.5. Relationships among Risk Scores, Clusters, Immune Cell Populations, and Clinicopathological Characteristics

For each sample, the number of cells among 22 types of immune cells (resting mast cells, regulatory T cells, M2 macrophages, CD8+ T cells, activated DCs, M0 macrophages, resting DCs, eosinophils, M1 macrophages, plasma cells, resting natural killer (NK) cells, CD4+ memory resting T cells, activated NK cells, monocytes, CD4+ naïve T cells, neutrophils, CD4+ activated memory T cells, memory B cells, gamma delta T cells, naïve B cells, follicular helper T cells, resting DCs, and activated mast cells) was estimated using the “CIBERSOFT” R package. Alternatively, the “ggpubr” R package was used to investigate the associations among the immune cells, risk score, clusters assessed by consensus clustering, and clinicopathological characteristics of patients with OSCC [22, 23].

The article "Identification of Nine M6A-Related Long Noncoding RNAs as Prognostic Signatures Associated with Oxidative Stress in Oral Cancer Based on Data from The Cancer Genome Atlas" was retracted in 2023. Reasons: signs of a paper mill; compromised peer review; unreliable results or conclusions.

### 2.6. Validation of Oxidative Stress-Related Genes in OSCC

Total RNA was isolated from OSCC tissues using TRIzol reagent (Sigma-Aldrich, St. Louis, MO, USA). Next, 2 *μ*g of RNA was isolated from each sample, and quantitative reverse transcription PCR was performed using the FastStart Universal SYBR ®Green Master (Roche, Germany) on an ABI QuantStudio5 Q5 real-time PCR System (Thermo Fisher Scientific, USA). cDNA was used as a template in a 20 *μ*L reaction volume (10 *μ*L of PCR mixture, 0.5 *μ*L of forward and reverse primers, 2 *μ*L of the cDNA template, and an appropriate volume of water). PCRs were performed as follows: cycling conditions began with an initial DNA denaturation step at 95°C for 30 s, followed by 45 cycles at 94°C for 15 s, 56°C for 30 s, and 72°C for 20 s. Each sample was examined in triplicate. Threshold cycle (CT) readings were collected and normalized to the glyceraldehyde 3-phosphate dehydrogenase (GAPDH) levels in all samples using the 2^-*ΔΔ*CT^ method. The mRNA expression levels were compared to those in precancerous tissue controls. The sequences of primer pairs for the target genes are shown in Table 1.

### 2.7. Statistical Analyses

R software (v4.0.5) was used to perform data analysis. Unless specified otherwise, statistical significance was considered at *p* < 0.05. The relationship between different clusters and their characteristics was analyzed using the chi-square test (*n* = 368). The relationship between the OS and individual factors was explored by univariate and multivariate Cox analyses (*n* = 368). Data visualization was performed using the “ggplot2” R package.

## 3. Results

### 3.1. Patient Characteristics

This work included 368 patients with OSCC. The average follow-up time was 888 days (1–5,480 days).

### 3.2. Prognostic M6A-Related lncRNAs in Patients with OSCC

Coexpression analysis was used to screen 1,080 M6A-related lncRNAs (Figure 1). Univariate Cox regression analysis identified 36 out of the total number of lncRNAs linked to OSCC prognosis.  Figure 2 presents the levels of lncRNAs in normal and OSCC samples as well as the hazard ratios (HRs).

The article "Identification of Nine M6A-Related Long Noncoding RNAs as Prognostic Signatures Associated with Oxidative Stress in Oral Cancer Based on Data from The Cancer Genome Atlas" was retracted in 2023. Reasons: signs of a paper mill; compromised peer review; unreliable results or conclusions.

### 3.3. Patient Clusters by Consensus Clustering

The consensus clustering distribution function (CDF) is displayed in Figures 3(a)–3(c), in which *k* = 2 to 9, along with the increment in the AUC of the CDF and the tracking plot in which *k* = 2 to 9, respectively. Based on the largest increment in the AUC and the association of the prognostic expression levels of M6A-correlated lncRNAs in the clusters, two OSCC clusters (*k* = 2, clusters 1 and 2) were subsequently identified (Figure 3(d)).

### 3.4. Clinical Characteristics and Pathway Analysis of the Different Clusters

Heat mapping showed that cluster 1 of patients was more advanced than the cluster 2 in terms of the T stage and the pathological grade (Figure 4(a)). Cluster 1 patients showed a dismal outcome (*p* < 0.001, Figure 4(b)), as shown by the KM survival analysis. Thereafter, we compared the expression and clinical characteristics of lncRNAs in the various clusters. In addition, the GSEA results suggested that compared with that in cluster 2 samples, certain pathways, such as oxidative stress, showed greater enrichment in cluster 1 samples (Figure 4(c)).

### 3.5. Predicting OSCC Prognosis Using the Risk Score Model, Based on 9-Key Prognostic M6A-Related lncRNAs

From the training group, we identified nine major M6A-related lncRNAs for prognosis. The risk score was determined as follows: risk score = ALMS1 − IT1∗0.627 + INC01106∗1.158 − AL603832.1∗0.280 − AC009120.3∗0.772 − AC008406.3∗0.270 − AC114730.3∗0.071 − LINC01305∗0.203 − AC037459.2∗0.130 − AC024267.4∗0.450. In both the test and training groups, the rates of survival of patients with high-risk diseases were lower (Figure 5(a)). The training group and the test group showed AUCs of the three-year OS curve of 0.75 and 0.69 (Figure 5(b)), respectively. In patients from the low-risk and high-risk score groups, the risk score could be distinguished accurately using survival state and risk plots (Figures 5(c) and 5(d)). In addition, for the survival of the two groups, the risk score was an independent factor, as revealed by the results of the univariate and multivariate analyses (Figures 6). Lastly, in populations with diverse clinicopathological characteristics, the prognostic value of the risk score was evaluated. Our data indicated that the prognosis in all categories, apart from that of patients with distant metastases, might be accurately distinguished using the risk score.

The article "Identification of Nine M6A-Related Long Noncoding RNAs as Prognostic Signatures Associated with Oxidative Stress in Oral Cancer Based on Data from The Cancer Genome Atlas" was retracted in 2023. Reasons: signs of a paper mill; compromised peer review; unreliable results or conclusions.

### 3.6. Relationship among Risk Scores, Clusters, Immune Cell Populations, Clinicopathological Characteristics, and Oxidative Stress-Associated Biomarker Expression

The risk score showed a negative correlation with the number of resting mast cells, naïve B cells, and plasma cells, but a positive correlation with the number of resting NK cells, follicular helper T cells, activated mast cells, and M2 macrophages (Figure 7). The risk score was higher for patients included in cluster 1, who had a poor prognosis, as compared to that for patients in cluster 2, who had a good prognosis. Additionally, patients with a high-risk score showed a more advanced AJCC stage and T stage than patients with a low-risk score (Figure 8). The relationship between the risk score and oxidative stress-associated biomarker expression indicated that the risk score could be affected by oxidative stress.

### 3.7. The Oxidative Stress-Related Gene Validation in OSCC Patients

The results of PCR showed that the biomarkers like HMOX1, NFE2L2, NOS2, NOS3, and TP53 which is associated with oxidative stress was validated that expressed higher in normal tissue (Figures 9 and 10).

## 4. Discussion

Despite recent advances in treatment methods, the 5-year survival in OSCC remains at approximately 60% owing to difficulties in early diagnosis and prognostic determination [24]. Recent studies have identified numerous effective OSCC biomarkers. Previously, based on the expression patterns of seven immunity-related genes, a prognostic model for OSCC was established [25]. We believe that the model developed in this study is critical for identifying useful and specific biomarkers for predicting OSCC outcomes.

Yang et al. developed a model for predicting prognosis based on 16 M6A-related lncRNAs in OSCC. However, only 164 patients were recruited for the study, and not all patients with OSCC who were included in TCGA databases were included. Concurrently, the study did not analyze the relationship between the lncRNAs and oxidative stress, a regulatory pathway involved in the development of oral cancer [26]. For the identification of new biomarkers of OSCC, we investigated the prognostic value of lncRNAs associated with M6A using TCGA data of 371 patients with OSCC and analyzed the relationship between these lncRNAs and oxidative stress pathways. Cox expression analysis was used to identify 1,080 M6A-related lncRNAs. Based on the findings of the univariate Cox regression analysis, 36 lncRNAs were found to be related to prognosis. Oxidative damage accumulates with aging in various species and in different tissues. RNA modification is mobilized to activate or inhibit stress-resistant signaling pathways [27]. Li et al. found that the activities of METTL3/METLL14, p21, and senescence-related *β*-galactosidase (SA-*β*GAL) increased significantly in oxidative damage-exposed HCT116 p53^−/−^cells, indicating that METTL3/METLL14 may trigger the p53-independent effect of aging in the oxidative damage response, which needs to be tested further [28]. Arsenite et al. stimulated human keratinocytes to induce reactive oxygen species (ROS) production, which thereby increased the WTAP, METTL14, and total M6A expression levels [29]. FTO induces oxidative stress and increases ROS levels by reducing the M6A methylation of peroxisome proliferator-activated receptor-gamma coactivator-1 alpha (PGC1*α*), an important regulator of mitochondrial metabolism that is also affected by the aging process, and increasing PGC1*α* mRNA translation efficiency. In our study, the M6A risk score was significantly associated with oxidative stress. This warrants an investigation of the underlying relationship.

The article "Identification of Nine M6A-Related Long Noncoding RNAs as Prognostic Signatures Associated with Oxidative Stress in Oral Cancer Based on Data from The Cancer Genome Atlas" was retracted in 2023. Reasons: signs of a paper mill; compromised peer review; unreliable results or conclusions.

Subsequently, depending upon the variations in the expression level of these prognostic M6A-associated lncRNAs, consensus clustering was used to divide the samples into two clusters. A more advanced pathological grade and T grade and worse outcomes were observed in patients in cluster 1, indicating that the prognosis of patients with OSCC could be accurately distinguished using the proposed method, and the M6A-related lncRNAs could influence the pathogenesis of OSCC. In addition, the findings of the GSEA suggested that “oxidative stress” was less enriched in cluster 2 than in cluster 1. The upregulation of the EMT pathway, which is associated with cancer cell invasion and metastasis, can increase the risk of cancer recurrence and reduce the survival rate [30]. Furthermore, EMT is involved in local recurrence, lymph node metastasis, and low survival rate among patients with OSCC [31]. However, the specific mechanism underlying this upregulation, and particularly its correlation with M6A-related lncRNAs, remains unclear.

Depending upon the results of the LASSO Cox regression analysis in the training group, nine prognostic hub M6A-related lncRNAs were filtered. Among these lncRNAs, ALMS1-IT1 was found to be associated with the poor prognosis of lung cancer and AC114730.3 with the good prognosis of bladder cancer [32, 33]. Reportedly, LINC01305 reduced the metastasis and invasion of ovarian and lung cancer by inhibiting EMT [34]. However, the mechanism underlying the action of the lncRNAs in OSCC, and the roles of AL603832.1, AC0091230.3, AC008406.3, AC037459.2, INC01106, and AC024267.4 in tumorigenesis remain unclear. In particular, their role in the initiation of OSCC requires further elucidation.

The article "Identification of Nine M6A-Related Long Noncoding RNAs as Prognostic Signatures Associated with Oxidative Stress in Oral Cancer Based on Data from The Cancer Genome Atlas" was retracted in 2023. Reasons: signs of a paper mill; compromised peer review; unreliable results or conclusions.

A risk score model was developed for the prediction of OSCC prognosis according to the coefficients of major prognosis-related M6A-associated lncRNAs and the FPKM values. We also compared the risk scores of the test and training groups. The risk score served as a reliable independent prognostic factor of OSCC, as indicated in the results obtained from the KM analysis, ROC curves, risk map analysis, and univariate and multivariate Cox regression analyses. Apart from that of patients with distant metastasis, the prognosis of populations with different clinicopathological characteristics could be predicted by the risk score. The risk score probably failed to distinguish among the prognosis of patients with distant metastasis because only eight patients were included in this category. In addition, patients who were present in the high-risk score group showed a more advanced T stage and AJCC stage and a shorter OS, whereas patients present in the low-risk cluster 2 showed a lower risk score than patients in the high-risk cluster 1. These results indicated that the key prognostic M6A-related lncRNAs identified in this study may be important for the initiation and progression of OSCC. Verification was performed to confirm the risk score accuracy and significance while predicting OSCC prognosis. To further confirm oxidative stress in patients with OSCC, we performed RT-PCR using tissues obtained from patients with OSCC to confirm the relationship between normal and OSCC patient groups. Prognostic data should be collected in the future to confirm the signature.

The risk score showed a negative correlation with the number of resting mast cells, naïve B cells, and plasma cells, but showed a positive correlation with the number of M2 macrophages, follicular helper T cells, NK cells, and activated mast cells. B cells are important in the host response to tumors, and naïve B cells inhibit tumor cell growth and promote good prognosis in prostate cancer and non-small-cell lung cancer [35, 36]. Alternatively, plasma cells can produce tumor-specific antibodies that can bind to tumor cells for inhibiting the activation of their complements and target proteins and/or for promoting antibody-dependent cytotoxicity [37]. The number of plasma cells has been associated with a good prognosis for lung cancer, liver cancer, and other tumors [38]. Similarly, the results of the present study indicated that plasma cells and naïve B cells are potentially associated with a good prognosis of OSCC. In contrast, mast cells undertake distinct functions in different tumors and can either promote or inhibit tumor growth [39]. Increased mast cell infiltration is linked to the poor prognosis of lung and colorectal cancer and good prognosis of breast and prostate cancer [40, 41]. The findings of a study on head and neck cancer suggested that activated mast cells were linked to a poor prognosis [42]. In the present study, the risk score showed a negative correlation with the number of resting mast cells but a positive correlation with the number of activated mast cells. These findings indicate that the latter can promote the growth of OSCC. Tumor-associated macrophages exhibit two distinct phenotypes: M1 (classically activated macrophages) and M2 (alternatively activated macrophages). M2 macrophages can contribute to tumor growth, angiogenesis, and immunosuppression [43]. The number of M2 macrophages is linked to the poor prognosis of patients with intrahepatic cholangiocarcinoma, renal cell carcinoma, and glioma [44, 45]. NK cells, which exhibit potent cytolytic activity, are important contributors to the host defense against tumors [46]. Although few studies have been conducted on the relationship between the number of resting NK cells and tumors, the number of resting NK cells was found to be positively correlated with the Gleason score in patients with prostate cancer, which indicates its correlation with prostate cancer malignancy [36]. The involvement of follicular helper T cells in the initiation and progression of tumors has been recognized. The formation and maintenance of the germinal center depend on follicular helper T cells, which represent the key cell type of the latter. These cells can promote B cell proliferation and somatic hypermutation and are linked to the poor prognosis of gastric and lung cancer [47]. In this study, the risk score showed a positive correlation with the number of M2 macrophages, follicular helper T cells, and resting NK cells, indicating the correlation of poor prognosis in OSCC with the population of these immune cell types. However, further research is necessary to understand how these cells interact during the initiation and progression of OSCC. The limitations of this study were the small sample size of adjacent normal tissues and the OSCC RNA sequence FPKM data. Thus, potential statistical errors could not be excluded. Further experiments are needed to explore the efficacy of the proposed prognostic model in the clinical environment to improve its reliability in terms of prognostic prediction in patients with OSCC. Additionally, no experiment was performed to confirm the interaction between the prognostic factors lncRNAs and M6A modulators in OSCC. Further investigation is necessary to confirm the relationship among M6A, oxidative stress, and OSCC.

The article "Identification of Nine M6A-Related Long Noncoding RNAs as Prognostic Signatures Associated with Oxidative Stress in Oral Cancer Based on Data from The Cancer Genome Atlas" was retracted in 2023. Reasons: signs of a paper mill; compromised peer review; unreliable results or conclusions.

In conclusion, to our knowledge, this is the first study to verify the expression and prognostic value of M6A-related lncRNAs in OSCC. The expression of M6A-related lncRNAs is closely related to the clinical characteristics and a poor survival rate in OSCC and can be used clinically to predict the prognosis of OSCC. Such findings will inform future investigations on the potential therapeutic targets of OSCC.

## Figures and Tables

**Figure 1:** Network of N6-methyladenosine (m6A) as red nodes and 1080 long noncoding RNAs (lncRNAs) as blue nodes (*n* = 371).

**Figure 2:** Identification of 36 prognostic N6-methyladenosine- (m6A-) relevant lncRNAs using univariate Cox regression analysis. (a) Heatmap of the prognostic expression m6A-relevant lncRNAs (*n* = 371). (b) Vioplot diagram of prognostic expression m6A-relevant lncRNAs (*n* = 371). (c) Forest plot and hazard ratio values obtained from univariate regression analysis (*n* = 368). ^∗^*p* < 0.05;  ^∗∗^*p* < 0.01;  ^∗∗∗^*p* < 0.01.

**Figure 3:** Consensus clustering of the OSCC TCGA cohort based on the levels of expression of 36 prognostic m6A-relevant lncRNAs (*n* = 368). (a) CDF for *k* = 2–9. (b) Increment in the area under the CDF curve for *k* = 2–9. (c) Tracking plot for *k* = 2–9. (d) Consensus matrix for the optimal value, i.e., *k* = 2. OSCC: oral squamous cell carcinoma; TCGA: The Cancer Genome Atlas; CDF: consensus clustering distribution function.

**Figure 4:** Varying prognoses, clinical characteristics, and pathways in different clusters. (a) Clinical characteristics and expression of lncRNAs in different clusters of patients with OSCC. (b) Kaplan-Meier OS curves for the different patients' clusters with OSCC. (c) Pathways enriched in comparison of cluster 1 (*n* = 325) with cluster 2 (*n* = 43). lncRNAs; long noncoding RNAs; OSCC: oral squamous cell carcinoma; OS: overall survival; ^∗^*p* < 0.05;  ^∗∗^*p* < 0.01;  ^∗∗∗^*p* < 0.01.

**Figure 5:** (a) The Kaplan-Meier analysis of patients present in the low-risk group and high-risk group in the test and training groups. (b) ROC curves of patients depicting high- and low-risk scores in the training (*n* = 184) and test groups (*n* = 184) (AUC = 0.75 and 0.69, respectively). (c, d) Risk plots and survival state of patients which present in the low-risk group and high-risk group in the test and training groups. ROC: receiver operating characteristic; AUC: area under the curve.

**Figure 6:** Results of the univariate and multivariate Cox regression analysis. (a) Training group of univariate Cox regression analysis. (b) Test group of univariate Cox regression analysis. (c) Training group of multivariate Cox regression analysis. (d) Test group of multivariate Cox regression analysis. *n* = 184 in both two group.

The article "Identification of Nine M6A-Related Long Noncoding RNAs as Prognostic Signatures Associated with Oxidative Stress in Oral Cancer Based on Data from The Cancer Genome Atlas" was retracted in 2023. Reasons: signs of a paper mill; compromised peer review; unreliable results or conclusions.

**Figure 7:** Relationship between the risk scores and immune cells (*n* = 368): (a) activated mast cells, (b) follicular helper T cells, (c) M2 macrophages, (d) naïve B cells, (e) plasma cells, (f) resting mast cells, and (g) resting NK cells.

**Figure 8:** Relationship between risk score, clusters, and clinicopathological characteristics (*n* = 368): (a) age, (b) Cluster, (c) gender, (d) grade, (e) tumor, (f) lymph node metastasis, (g) distant metastasis, and (h) stage.

**Figure 9:** Relationship between risk score and oxidative stress expression (*n* = 184 in both two group).

**Figure 10:** The expression of oxidative stress related genes (*n* = 6).

**Table 1:** Primer pairs for the target genes.

Gene	Forward primer sequence (5-3)	Reverse primer sequence (5-3)
NOS3	GCCGGAACAGCACAAGAGTTA	CCCTGCACTGTCTGTGTTACT
NFE2L2	AGGTTGCCCACATTCCCAAA	ACGTAGCCGAAGAAACCTCA
TP53	ACCTATGGAAACTACTTCCTGAAA	CTGGCATTCTGGGAGCTTCA
NOS2	GCTTTGTGCGAAGTGTCAGT	TTGTGCTGGGAGTCATGGAG
HMOX1	AGTTCAAGCAGCTCTACCGC	GCAACTCCTCAAAGAGCTGGAT
GAPDH	AATGGGCAGCCGTTAGGAAA	GCCCAATACGACCAAATCAGAG

## Data Availability

The datasets used and/or analyzed during the current study are available from the corresponding author on reasonable request.

## Abbreviations

M6A: N6-methyladenosine
lncRNA: Long noncoding RNA
OSCC: Oral squamous cell carcinoma
TCGA: The Cancer Genome Atlas
GSEA: Gene set enrichment analysis
OS: Overall survival
AJCC: American Joint Committee on Cancer
HOTAIR: HOX transcript antisense intergenic RNA
LASSO: Least absolute shrinkage and selection operator
KM: Kaplan-Meier
DCs: Dendritic cells
NK: Natural killer
ROC: Receiver operating characteristic
CDF: Cumulative distribution function
AUC: Area under the curve.
